# Long-Term Elevated Siglec-10 in Cerebral Spinal Fluid Heralds Better Prognosis for Patients with Aneurysmal Subarachnoid Hemorrhage

**DOI:** 10.1155/2022/5382100

**Published:** 2022-09-21

**Authors:** Sen Gao, Xun-Zhi Liu, Ling-Yun Wu, Zheng Peng, Xiang-Xin Chen, Han Wang, Yue Lu, Zong Zhuang, Qian Tan, Chun-Hua Hang, Wei Li

**Affiliations:** ^1^Department of Neurosurgery, Nanjing Drum Tower Hospital, The Affiliated Hospital of Nanjing University Medical School, Nanjing, China; ^2^Department of Burns and Plastic Surgery, Nanjing Drum Tower Hospital, The Affiliated Hospital of Nanjing University Medical School, Nanjing, China

## Abstract

The presence of aneurysmal subarachnoid hemorrhage (aSAH) is usually accompanied by excessive inflammatory response leading to damage of the central nervous system, and the sialic acid-binding Ig-like lectin 10 (Siglec-10) is a recognized factor being able to modify the inflammatory reaction. To investigate the potential role of Siglec-10 in aSAH, we collected the cerebrospinal fluid (CSF) of control (*n* = 11) and aSAH (*n* = 14) patients at separate times and measured the Siglec-10 concentration utilizing the enzyme-linked immunosorbent assay (ELISA) and evaluated the alterations of GOS and GCS during the disease process. In accordance with the STROBE statement, results showed that Siglec-10 in CSF rose quickly in response aSAH attack and then fell back to a slightly higher range above baseline, while it remained at relative high concentration and last longer in several severely injured patients. In general, higher Siglec-10 expression over a longer period usually indicated a better clinical prognosis. This prospective cohort study suggested that Siglec-10 could possibly be used as a biomarker for predicting prognosis of aSAH due to its ability to balance aSAH-induced nonsterile inflammation. Additionally, these findings might provide novel therapeutic perspectives for aSAH and other inflammation-related diseases.

## 1. Introduction

Aneurysmal subarachnoid hemorrhage (aSAH) refers to extravasation of blood into the subarachnoid space caused by the aneurysm rupture, which is the most common cause for SAH [1, 2]. After aSAH attack, a cascade of pathophysiological changes including inflammation, ionic disbalance, oxidative stress, ischemia, and hypoxia would sabotage central nervous system [3]. Unfortunately, despite advanced progress in surgical technique and intensive caring capacity, SAH-related mortality rate still remained around 8% to 67% with high morbidity [4–7]. Therefore, there is an urgent demand to make clear the pathological mechanism of and find beneficial factors promoting better clinical prognosis for aSAH.

The sialic acid-binding Ig-like lectins (Siglecs) are members of the immunoglobulin superfamily expressed on the cell surface and were recognized as negative regulator in modulating innate and adaptive immune functions [8, 9], which depends on so-called immunoreceptor tyrosine-based inhibitory motifs (ITIMs) [10, 11]. Siglec-10 is a member of the Siglec family working upstream of ITIMs. It is widely expressed on human leucocytes, including B cells, eosinophils, monocytes, dendritic cells, T cells, and NK cells [12–16]. Studies have shown that Siglec-10 is embed with an important role in regulating the immune balance. For example, the interaction of Siglec-10 and CD24 could reduce the damage-associated molecular patterns- (DAMPs-) induced inflammatory response via inhibiting the activation of high mobility group box 1 (HMGB1) and NF-*κ*B [17–20]. The interaction between Siglec-10 expressed on human DCs and pseudaminic acid can promote the expression of IL-10 through MyD88 and p38/MAPK signaling pathway to boost anti-inflammatory function [21]. Several other reports have also validated its immune-modulating influence on the inflammatory microenvironment [22–25]. Research on oncology indicates that tumors could evade immunological surveillance through inhibiting NK cells and T cells and repressing tumour-killing capacity of macrophages with high Siglec-10 expression [26, 27]. In contrast, blocking macrophage Siglec-10 can increase macrophage-mediated phagocytosis [28]. Additionally, Siglec-10 also plays a role in the establishment of immune tolerance [29].

Given that inflammatory response is an important pathological process of aSAH, excessive unresolved inflammation could cause considerable damage to central nervous system [20], thus Siglec-10, as an anti-inflammatory factor, may affect the recovery of aSAH patients by via balancing proper inflammation, while this has yet not been validated in vivo or in vitro. To test this hypothesis, we conducted this clinical experiment to figure out if Siglec-10 is involved in the pathophysiological process after aSAH and the potential relationship between cerebrospinal Siglec-10 content and the prognosis of patients.

## 2. Materials and Methods

All the methods used for human trials were made in line with the Helsinki Declaration and approved by the medical institutional review board (no. 2020-041-01) at Nanjing Drum Tower Hospital. All clinical samples were obtained with the written informed consent of the patients or their families.

### 2.1. Patient Selection

The selection criteria of the experimental group were described as below: (1) diagnosed as aSAH by admission CT scan; (2) Hunt and Hess scale (HH) 1 or 2, while more severely injured patients were not enrolled to avoid iatrogenic damage; (3) no other CNS disease; (4) the experimental group received interventional treatment of endovascular embolization with coils within two days after aSAH; (5) no diabetes, malignant tumors, connective tissue diseases, or other systemic diseases. A flow diagram for the inclusion of aSAH patients in this study is presented in Figure 1. The patients' condition evaluation of the experimental group was shown in Table 1. The control group was obtained from patients who undergone surgeries with lumbar subdural anaesthesia with no SAH or any other CNS disease.

### 2.2. Sample Collection and Detections

The cerebrospinal fluid (CSF) samples (5 mL per sample) in the experiment was obtained from the experimental group (*n* = 14) and the control group (*n* = 11) by lumbar puncture or external ventricular drainage. CSF of the experimental group was extracted from patients on day 3, day 7, and day 9 after aSAH. And CSF from control group patients was set as control. All clinical samples were centrifuged (3000 g, 5 min) in a sterile tube, and the supernatant was taken and stored at -80°C before test.

The enzyme-linked immunosorbent assay (ELISA) was then conducted to determine the protein levels of Siglec-10 in CSF after enough samples were collected. We used the commercial human ELISA kit (cat# MBS2509371, MyBioSource) in this study according to the manual.

### 2.3. Assessment of Recovery Status and Grouping

We evaluated the Glasgow Outcome Scale (GOS) and Glasgow Coma Scale (GCS) of patients on admission, day 3, day 7, day 9, and at discharge. All patients were admitted and received interventional therapy within two days after aSAH.

To explore the correlation between Siglec-10 and the prognosis of patients, a feasible method was to allocate patients on the basis of GOS score alteration-patients with better GOS amelioration were assigned to one group and the others to another. Then, the Siglec-10 levels variance between different groups were compared. As shown in Table 2, only one patient's GOS deteriorated on day 3 and all patients' GOS increased to 5 points at discharge, making data not suitable for being grouped by GOS score alterations day 3 or at discharge. Still, we can make reasonable groupings based on GOS score changes on day 7 and day 9. In this way, patients were divided into GOS-elevated and unchanged groups. Another way to investigate their correlation was to analyze whether the GOS at admission was related to Siglec-10 levels in the following days.

The GCS of the patients is shown in Table 3. It was difficult to group by score changes to make qualitative analysis because only one patient among the patients had no full GCS score on admission and had no GCS change on day 3. Meanwhile, all patients got full 15 points since day 7. Considering the potential protective effects of Siglec-10, we directly analyzed the relationship between Siglec-10 levels and GCS changes, including the correlation between Siglec-10 levels on day 3 and GCS changes on day 3 or day 7 and the correlation between Siglec-10 levels on day 7 and GCS changes on day 7. Besides, the correlation between GOS at admission and Siglec-10 levels on the following days was also examined.

### 2.4. Data Analysis

We used GraphPad Prism7.0 to analyze the data. One-way analysis of variance with Dunnett's T3 and Tukey's post hoc tests was used when comparing three or more groups. Unpaired Student's *t*-test was used when comparing two groups. Pearson correlation coefficient was used to evaluate the simple correlation between continuous variables. *P* < 0.05 was considered to be statistically significant. Data were expressed as mean ± SEM.

## 3. Results

### 3.1. Siglec-10 Levels in CSF Increased Rapidly after aSAH

We observed that patients in different groups and at different time points had different Siglec-10 levels (Figure 2). The Siglec-10 expression in the control group was at a low level. Meanwhile, Siglec-10 of aSAH patients quickly peaked on day 3 (*P* < 0.05) and then plateaued since day 7, though not as high as day 3 but still higher than that of the control group (*P* < 0.05).

### 3.2. Longer Maintenance of High-Level Siglec-10 Indicated Better GOS Improvements

Whether Siglec-10 played a role in the process of aSAH can be clarified by group comparison. When groups were divided according to GOS alteration on day 7, there was no significant difference in Siglec-10 levels at any given time point (Figure 3(a)). While on day 9, different groups showed a significant difference of Siglec-10 levels on day 7 (Figure 3(b), *P* < 0.05), but not on day 3 or day 9. This meant that the interblock difference could not be observed by the time of Siglec-10 expression peak until day 7, indicating that the difference observed on day 7 was more likely a result of different Siglec-10 expression fluctuations. In addition, regardless of the grouping, there is no difference in age between groups (Table 4).

There was not only a qualitative but also a quantitative relationship between Siglec-10 expression level and GOS changes. Our results showed that the GOS score alterations from admission to day 9 was positively correlated with the Siglec-10 expression on day 7 (Figure 4(a), *r* = 3.597, *P* < 0.05). The GOS score variation between admission and discharge conformed to the same pattern (Figure 4(b), *r* = 3.178, *P* < 0.05). As the level on day 7 reflected whether Siglec-10 maintained high concentration for a longer time, it can be summarized that the longer the Siglec-10 can be maintained at a high level, the better the prognosis seemed to be in the following days.

### 3.3. The High-Level Siglec-10 Lasted Longer in Patients with Relatively Severe Injuries

Further, we analyzed the relationship between Siglec-10 levels and the severity of patients on admission, which is reflected by GOS and HH. The results showed that Siglec-10 levels on day 7 was significantly correlated with the GOS on admission. Patients with lower GOS on admission had higher Siglec-10 levels on day 7 (Figure 5(b), *r* = −3.178, *P* < 0.05). No such phenomenon was observed on day 3 (Figure 5(a)) or day 9 (Figure 5(c)).

There were similar results in HH. Compared to HH1, HH2 patients had even higher levels of Siglec-10 on day 7 (Figure 6(b), *P* < 0.05).

### 3.4. Siglec-10 Was Not Significantly Related to the Changes of GCS

The association between GCS and Siglec-10 could not be clearly observed. On the one hand, there was no significant correlation between the GCS at admission and Siglec-10 levels, whether on day 3 (Figure 7(a)), day 7 (Figure 7(b)), or day 9 (Figure 7(c)). On the other hand, there was no correlation between the changes of GCS on day 3 and Siglec-10 levels on day 3 (Figure 7(d)), or the changes of GCS on day 7 and Siglec-10 levels on day 3 (Figure 7(e)) or day 7 (Figure 7(f)).

## 4. Discussion

After binding to its ligand, the tyrosine residing in the ITIM domain of Siglec-10 will be phosphorylated and serves as a binding site for proteins containing the SH2 domain (SHP phosphatase for instance). Which would then lead to the dephosphorylation of cytoplasmic proteins and therefore downregulate the downstream signaling pathways [30]. By negatively regulating the resultant inhibition of NF-*κ*B, Siglec-10 can retain the damage of DAMP-related inflammatory response [17]. Through MyD88 and p38 MAPK signaling pathways, Siglec-10 can increase the expression of IL-10 to promote anti-inflammatory function [21]. Siglec-10 can also inhibit the function of NK cells and T cells or interact with HSP70, HSP90, and VAP1 to repress inflammation [17, 22]. There are many consistent researches in the field of aSAH, such as MyD88/NF-*κ*B pathway, HMGB1 and DAMPs [31–34]. Our results showed that Siglec-10 rose instantly and soon peaked after aSAH and remained at a high concentration afterwards, indicating that Siglec-10 did participate in the pathophysiological process after aSAH. Still, these results alone cannot characterize the comprehensive role of Siglec-10 due to the complex pathological process as well as numerous cytokines or inflammatory mediators released during this process, so we conducted the analysis below.

In our experiment, patients with Siglec-10 maintained at high levels for a longer period seemed to have better prognosis, which was approved by both qualitative and quantitative analysis. This finding confirmed that high-level and long-term Siglec-10 in CSF was associated with better outcomes for aSAH patients. Another potential role of Siglec-10 was that expression and duration of CSF Siglec-10 expression seemed to be related with severity on admission. Upon exposing to damage, the host initiates defensive mechanisms in react to such stress. Naturally, the heavier the host was injured, the prompter protective reactions would be provoked. This phenomenon is consistent with the performance of Siglec-10 in our experiment. Another noteworthy point is that why Siglec-10, generally regarded as a membrane-tethered receptor, appeared in CSF. We suspect that it might be the result of blood-brain barrier breaking down and the subsequent infiltration of inflammatory cells expressing Siglec-10 into the CSF. This also explains why the Siglec-10 levels of the control group were relatively low.

Interestingly, we could find that Figures 4(b) and 5(b) have the symmetrical correlation coefficients. The reason is that the GOS of patients all reached a perfect score of 5 at discharge. Presume that if not all patients had a full score when they get discharged, then Figure 5(b) would remain the same, but Figure 4(b) would show a different correlation coefficient. Furthermore, if there were data of more time points such as day 8, day 10, and day 11, new results would support our argumentation more strongly.

As for the analysis of GCS, regrettably, no correlation was found, and the explanation was quite complex. For example, though both scales were used to assess aSAH patients, GCS tends to characterize the degree of consciousness, while GOS is the more accurate descriptor of prognosis. Besides, patients in our experiment were mildly injured with almost all GCS above 12 points, which might result in less significant comparisons; most patients had recovered to the full score on day 3, causing difficulties in the grouping. These biases could be possibly reduced by recruiting more severely injured patients, increasing the frequency of evaluating GCS, and expanding the sample size. Speaking of the limits, future research should be carried out more complicated experiments combined with other factors that may affect the prognosis, such as vasospasm, hydrocephalus, location, and size of the ruptured aneurysm, so that the results will be more accurate and more likely to reflect the characteristics of Siglec-10. Whether upregulating Siglec-10 exogenously could promote recovery also can be included in our future research.

## 5. Conclusions

Altogether, the present study suggested that the Siglec-10 expression level in CSF boosted in response to aSAH quickly peaked and then fall back to a stable range slightly higher above normal limit. Patients who were relatively severely injured are more likely to maintain high-level Siglec-10 for a longer period compensatorily. In general, having high-level and long-term Siglec-10 expression usually indicates superior prognosis, which is probably due to the anti-inflammatory effects avoiding the host's excessive inflammatory response to damage. The potential explanation might be that the anti-inflammatory function of Siglec-10 could avoid excessive host defense and ameliorating secondary damages. The exploration of the role of Siglec-10 in aSAH may provide a new predictive biomarker or new treatment alternatives for aSAH and other inflammation-related diseases.

## Figures and Tables

**Figure 1:** Flow diagram of patient selection.

**Figure 2:** Siglec-10 in CSF measured by ELISA. The protein levels of Siglec-10 in CSF of patients on the 3rd, 7th, and 9th days after the occurrence of aSAH and the control group. The Siglec-10 levels on day 3 show a significant difference with other days (*P* < 0.05 versus indicated groups). All data were expressed as the mean ± SEM.

**Figure 3:** Differences in Siglec-10 levels between GOS-elevated and unchanged groups. (a) Grouped according to whether GOS was higher than admission on day 7, there was no significant difference in Siglec-10 content at each time point. (b) Grouped according to whether GOS was higher than admission on day 9, the Siglec-10 levels in CSF on day 7 showed a difference (*P* < 0.05 versus indicated groups). All data were expressed as the mean ± SEM.

**Figure 4:** Relationship between Siglec-10 levels on day 7 and changes of GOS on the following days. The relationship between the Siglec-10 levels on day 7 and the changes of GOS on day 9 (a) and at discharge (b) was significantly correlated.

**Figure 5:** Relationship between GOS at admission and Siglec-10 levels at various time points. The Siglec-10 levels on day 7 was significantly correlated with GOS at admission (b). There was no significant correlation between GOS at admission and Siglec-10 levels on day 3 (a) or day 9 (c).

**Figure 6:** Differences in Siglec-10 levels of patients with different HH. The Siglec-10 levels on day 7 between HH1 and HH2 patients show a difference (*P* < 0.05 versus indicated groups). All data were expressed as the mean ± SEM.

**Figure 7:** Relationship between Siglec-10 levels at different time points and the GCS levels and changes. (a) Relationship between GCS at admission and Siglec-10 levels on day 3. (b) Relationship between GCS at admission and Siglec-10 levels on day 7. (c) Relationship between GCS at admission and Siglec-10 levels on day 9. (d) Relationship between the changes of GCS on day 3 and Siglec-10 levels on day 3. (e) Relationship between the changes in GCS on day 7 and Siglec-10 levels on day 3. (f) Relationship between the changes in GCS on day 7 and Siglec-10 levels on day 7.

**Table 1:** Injury status of aSAH patients.

Case	Gender	Age	Aneurysm location	Hunt-Hess	GCS on admission	GOS on admission
1	Male	42	V4 segment of left vertebral artery	II	13	3
2	Female	57	Anterior communicating artery	II	15	3
3	Female	57	Right posterior communicating artery	II	13	3
4	Male	49	The bifurcation of right middle cerebral artery	I	15	4
5	Female	51	Anterior communicating artery	II	12	3
6	Female	76	Anterior communicating artery	I	15	4
7	Female	46	Posterior communicating artery	II	12	3
8	Female	48	Apex of basilar artery	II	15	3
9	Female	65	Left anterior choroidal artery	I	15	4
10	Male	52	The bifurcation of middle cerebral artery	I	15	4
11	Female	65	Left posterior communicating artery	I	15	5
12	Female	49	Right posterior communicating artery	I	13	4
13	Male	68	Right anterior choroidal artery	II	13	3
14	Female	45	Apex of basilar artery	I	15	4

**Table 2:** GOS of aSAH patients at different time points.

Case	Admission	Day 3	Day 7	Day 9	Discharge
1	3	3	3	4	5
2	3	3	4	4	5
3	3	3	3	4	5
4	4	3	4	4	5
5	3	3	4	4	5
6	4	3	4	4	5
7	3	3	4	4	5
8	3	3	4	4	5
9	4	3	4	4	5
10	4	4	4	5	5
11	5	5	5	5	5
12	4	4	4	4	5
13	3	3	4	4	5
14	4	5	5	5	5

**Table 3:** GCS of aSAH patients at different time points.

Case	Admission	Day 3	Day 7	Day 9	Discharge
1	13	13	15	15	15
2	15	15	15	15	15
3	13	15	15	15	15
4	15	15	15	15	15
5	12	12	15	15	15
6	15	15	15	15	15
7	12	14	15	15	15
8	15	15	15	15	15
9	15	15	15	15	15
10	15	15	15	15	15
11	15	15	15	15	15
12	13	15	15	15	15
13	13	15	15	15	15
14	15	15	15	15	15

**Table 4:** Differences in age between GOS-elevated and unchanged groups.

Way to group	Average age of GOS-elevated group	Average age of unchanged group	*P*
By day 7	56.88	52.50	0.4425
By day 9	51.78	60.80	0.1097

## Data Availability

Data of this study is available on request.
